# Early Prediction of Cerebral Computed Tomography under Intelligent Segmentation Algorithm Combined with Serological Indexes for Hematoma Enlargement after Intracerebral Hemorrhage

**DOI:** 10.1155/2022/5863082

**Published:** 2022-06-14

**Authors:** Wenting Xu, Weizhou Tang, Liangqun Wu, Qianzhu Jiang, Qiyuan Tian, Ce Wang, Lina Lu, Ying Kong

**Affiliations:** ^1^Second Affiliated Hospital, Heilongjiang University of Chinese Medicine, Harbin, 150001 Heilongjiang, China; ^2^First Affiliated Hospital, Heilongjiang University of Chinese Medicine, Harbin, 150040 Heilongjiang, China; ^3^School of Clinical Medicine, Chengdu University of TCM, Chengdu, 610036 Sichuan, China

## Abstract

The aim of this study was to explore the application value of brain computed tomography (CT) images under intelligent segmentation algorithm and serological indexes in the early prediction of hematoma enlargement in patients with intracerebral hemorrhage (ICH). Fuzzy *C*-means (FCM) intelligence segmentation algorithm was introduced, and 150 patients with early ICH were selected as the research objects. Patient cerebral CT images were intelligently segmented to assess the diagnostic value of this algorithm. According to different hematoma volumes during CT examination, patients were divided into observation group (hematoma enlargement occurred, *n* = 48) and control group (no hematoma enlargement occurred, *n* = 102). The predicative value of hematoma enlargement after ICH was investigated by assessing CT image quality and measuring intracerebral edema, hematoma volume, and serological indicators of the patients of the two groups. The results demonstrated that the sensitivity, specificity, and accuracy of CT images processed by intelligence segmentation algorithm amounted to 0.894, 0.898, and 0.930, respectively. Besides, early edema enlargement and hematoma of patients in the observation group were more significant than those of patients in the control group. Relative edema volume was 0.912, which was apparently lower than that in the control group (1.017) (*P* < 0.05). In terms of CT signs of ICH patients, the incidence of blend sign, low density sign, and stroke of the observation group was evidently higher than those of the control group (*P* < 0.05). Besides, absolute lymphocyte count (ALC) and hemoglobin (HGB) concentration of the patients in the observation group were 6.23 × 109/L and 6.29 × 109/L, respectively, both of which were higher than those of the control group (6.08 × 109/L and 4.25 × 109/L). Neutrophil to lymphocyte ratio (NLR) was 0.99 × 109/L, which was apparently lower than that in the control group (1.43 × 109/L) (*P* < 0.05). To sum up, cerebral CT images processed by FCM algorithm showed good diagnostic effect on ICH and high clinical values in the early prediction of hematoma among ICH patients.

## 1. Introduction

Intracerebral hemorrhage (ICH) is a type of stroke accounting for about 13%, and it is the localized hemorrhage in surrounding tissues caused by the rupture of cerebral arteries [1]. ICH can be caused by a variety of causes, including head trauma, hypertension, aneurysm, vascular anomaly, blood diseases or bleeding disorders, liver diseases, and brain tumors [2, 3]. The symptoms of ICH are complex and diverse and are related to the bleeding site, volume, speed, size of the hematoma, and the patient's physical condition [4]. In addition, some patients will experience early hematoma enlargement after ICH, which can be observed in patients within 24 hours of the occurrence. It usually is manifested as an increase in hematoma volume. If the increase is more than one-third of the basic standard, it can be regarded as significant early hematoma enlargement [5, 6]. The current researches showed that 40% of ICH patients will experience early hematoma enlargement, and this symptom may be one of the key predictors of the prognosis of ICH patients. It usually occurs within 6 hours after the onset, and it also may occur within 24 hours; the probability of early hematoma enlargement is greatly reduced after 24 hours. Therefore, it is very important to pay attention to the changes of the patients' condition in the super early stage of the disease and to conduct computed tomography (CT) follow-up in time [7]. Hematoma enlargement after ICH often indicates a poor prognosis for patients, accompanied with aggravation of neurological damage; that is to say, the clinical symptoms of patients may be aggravated, and patients even suffer from disturbance of consciousness. Some patients with early hematoma enlargement may experience early death. Therefore, attention to early hematoma enlargement plays a very important role in the diagnosis and treatment of cerebrovascular disease [8].

Imaging examination is an important method for the diagnosis of ICH, and cerebral CT examination is the gold standard for the diagnosis of early ICH. At present, clinical imaging examination is a common method for diagnosing and understanding the etiology of ICH [9]. Plain CT scanning can quickly and accurately display the location of ICH, the amount of hemorrhage, mass effect, whether it has broken into the ventricle or the subarachnoid space, and the surrounding brain tissue damage. It is the preferred imaging method for patients with suspected stroke. Contrast media extravasation into the hematoma can be observed under enhanced CT scanning, which is important evidence suggesting a high risk of hematoma enlargement. Perfusion CT can reflect the hemodynamic changes of brain tissues after ICH and can be used to know the blood perfusion around the hematoma [10]. Reports in recent years have pointed out that there is a significant correlation between the enlargement of hematoma in ICH patients and the imaging features such as leakage sign, swirl sign, spot sign, black hole sign, and blend sign in CT imaging and CT angiography (CTA). Such a correlation can be used as one of the reliable indexes for the diagnosis of hematoma enlargement in patients with ICH [11]. In addition, several works have suggested that serological indexes are potential predictors of hematoma enlargement in patients with ICH [12].

At present, there are multiple reports on the diagnostic values of CT image characteristics in the prediction of hematoma enlargement among clinical ICH patients. However, original cerebral CT affect the doctor's clinical diagnosis and recognition of symptoms due to some problems with image quality, such as noise and artifact [13, 14]. In recent years, a great number of scholars introduced specific models or research results from other fields into medical image segmentation fields to solve the problem that traditional image segmentation algorithm could not process complex images with high precision. Besides, they designed various emerging algorithms, including clustering-based algorithm, wavelet transform segmentation algorithm, and artificial network segmentation algorithm. The typical representatives of clustering algorithm include *K*-means clustering algorithm and fuzzy *C*-means (FCM) algorithm. *K*-means clustering algorithm is easy to be implemented. However, the number of clusters and the initial value need to be specified in advance. Besides, the algorithm is sensitive to noise. FCM algorithm shows fuzzy clustering property. Compared with other algorithms, FCM algorithm is more suitable for the segmentation of CT images. It was pointed out in previous studies that FCM algorithm-based showed good precision, peak signal to noise ratio (PSNR), and mean square error (MSE) in the prediction of tumor tissues of lung CT images of patients with lung cancer. Consequently, the diagnostic accuracy of patients could be significantly improved [15].

Hence, it was expected that an intelligence segmentation algorithm was introduced into the diagnosis of cerebral CT images of ICH patients and patient serological indicators were combined to predict hematoma enlargement of ICH patients and assess the predictive values of two methods. Based on the traditional postoperative prevention of ICH patients, the predictive values of hematoma enlargement characteristics among patients in the postoperative development of disease among ICH patients were expected to be further assessed.

## 2. Materials and Methods

### 2.1. Research Objects

A total of 150 patients with early ICH were included as the research objects, who were diagnosed in the hospital from February 2019 to May 2021. There were 69 males and 81 females, with the age of 34-83 years and the average age of 58.62 ± 10.27 years. All patients underwent cerebral CT examination, including the initial examination within 6 hours of ICH and the reexamination 24 hours after the initial examination. Patient CT image data was measured quantitatively. The quantitative measurement indicators of CT images included edema volume, hematoma volume, and relative edema volume. CT images were compared. Patients suffering from hematoma enlargement were included in the observation group (*N* = 48 cases), and the group without hematoma enlargement was labeled as the control group (*N* = 102 cases). All procedures had been approved by the ethics committee of the hospital, and the objects included signed the informed consents.

The inclusion criteria for the patients were follows. The patients met the diagnostic criteria for early ICH and have the first occurrence of ICH. The hospitalization time after the occurrence was less than 6 hours, as the initial CT examination within 6 hours and the follow-up CT images after 24 hours were included. The exclusion criteria for patients were as follows. The ICH belonged to traumatic hemorrhage caused by traumatic brain injury. The ICH in patients was a secondary bleeding caused by aneurysm, vascular malformation, cerebral infarction, brain tumor, etc. The hematoma flew into the ventricles.

### 2.2. Cerebral CT Scanning Equipment and Parameters

The included cerebral CT plain scan imaging examination instrument was 16-slice spiral CT scanner. The main instrument parameters included slice thickness (6 mm), slice interval (6 mm), tube current (300 mA), and tube voltage (120 kV).

### 2.3. Cerebral CT Image Model of Patients with ICH under Intelligent Segmentation Algorithm

The fuzzy *C*-means (FCM) intelligent segmentation algorithm [16] was used to intelligently segment brain CT images of patients with ICH. This algorithm is a soft clustering algorithm with the attribute of fuzzy clustering. It could require the similarity of objects in the same cluster during the clustering process and finally divide the objects into the cluster with the largest degree of membership [17, 18]. The following was the construction process of the algorithm.

First, the objective function of the FCM algorithm was *H*(*A*, *B*), the number of clusters was *Q*, and *n* represented the fuzzy factor. Then, the mathematical expression of the objective function *H*(*A*, *B*) could be expressed as equation (1). The Euclidean distance from the specific sample point *u*_*s*_ to the cluster center *b*_*s*_ was adopted and represented by *d*_*zs*_, which was expressed as equation (2). The membership degree of the sample point (*s*) to the specific cluster (*z*) was represented by *μ*_*sz*_^*n*^, whose value satisfied equation (3).

(1) $$\begin{array}{c} H\left(A,B\right)=\overset{Q}{\underset{s=1}{\sum }}\overset{w}{\underset{z=1}{\sum }}\left(\mu_{\text{sz}}^{n}{\left(\sqrt{\overset{w}{\underset{z=1}{\sum }}{\left(u_{z}-b_{s}\right)}^{2}}\right)}^{2}\right), \end{array}$$

(2) $$\begin{array}{c} d_{zs}=\left\|u_{z}-b_{s}\right\|, \end{array}$$

(3) $$\begin{array}{c} \left\{\begin{array}{cc} 0\leq \mu_{sz}^{n}\leq 1, & s=1,2,\cdots ,w,\\ \overset{Q}{\underset{s=1}{\sum }}\mu_{sz}=1, & 1\leq s\leq Q,\\ 0\leq \overset{w}{\underset{z=1}{\sum }}\mu_{sz}\leq w, & 1\leq z\leq w. \end{array}\right. \end{array}$$

After that, the Lagrange multiplier [19] *λ*_*z*_(*z* = 1, 2, ⋯, *w*) was introduced into the objective function, to reconstruct the objective function. The transformation function *K*(*A*, *B*, *λ*) could be obtained, and its mathematical expression was shown as equation (4). By taking the partial derivative of equation (4), equation (5), equation (6), and equation (7) could be worked out.

(4) $$\begin{array}{c} K\left(A,b_{1}\cdots b_{Q},\lambda_{1}\cdots \lambda_{w}\right)=\overset{w}{\underset{z=1}{\sum }}\lambda_{z}\overset{Q}{\underset{s=1}{\sum }}\left(\mu_{sz}-1\right)+\overset{w}{\underset{z=1}{\sum }}\overset{Q}{\underset{s=1}{\sum }}\left(\mu_{sz}^{n}{\left(\sqrt{\overset{w}{\underset{z=1}{\sum }}{\left(u_{z}-b_{s}\right)}^{2}}\right)}^{2}\right), \end{array}$$

(5) $$\begin{array}{c} \frac{\partial K}{\partial \lambda }=\overset{Q}{\underset{s=1}{\sum }}\mu_{sz}-1, \end{array}$$

(6) $$\begin{array}{c} \frac{\partial K}{\partial \mu_{sz}}=n{\left(\mu_{sz}\right)}^{n-1}{\left(d_{zs}\right)}^{2}-\lambda_{z}, \end{array}$$

(7) $$\begin{array}{c} \frac{\partial K}{\partial b_{s}}=\overset{w}{\underset{z=1}{\sum }}{\left(\mu_{sz}\right)}^{n}u_{z}-b_{s}\overset{w}{\underset{z=1}{\sum }}{\left(\mu_{\text{sz}}\right)}^{n}. \end{array}$$

Since equations (5), (6), and (7) satisfied equation (8), the expressions of *b*_*s*_ and *μ*_*sz*_^*n*^ were derived as equation (9) and equation (10), respectively.

(8) $$\begin{array}{c} \left\{\begin{array}{c} \frac{\partial K}{\partial \mu_{sz}}=0,\\ \frac{\partial K}{\partial \lambda }=0,\\ \frac{\partial K}{\partial b_{s}}=0, \end{array}\right. \end{array}$$

(9) $$\begin{array}{c} b_{s}=\frac{\sum_{z=1}^{w}{\left(\mu_{sz}\right)}^{n}u_{z}}{\sum_{s=1}^{Q}{\left(\mu_{sz}\right)}^{n}}, \end{array}$$

(10) $$\begin{array}{c} b_{s}=\frac{1}{\sum_{W=1}^{Q}{\left(d_{zs}/d_{zW}\right)}^{2/\left(n-1\right)}}. \end{array}$$

### 2.4. Evaluation of Cerebral CT Image Quality in Patients with ICH under Artificial Intelligent Segmentation Algorithm

The dataset used was the BraTs2017 dataset, and the experimental environment adopted the Titanx device with 12G video memory for training set. The sensitivity, specificity, accuracy (Dice), and indexes were introduced to evaluate the quality of cerebral CT images of ICH patients, as the images were processed by intelligent segmentation algorithm. The sensitivity, specificity, and Dice were calculated by

(11) $$\begin{array}{c} \text{Sensitivity}=\frac{\left|a\cap c\right|}{\left|a\right|}, \end{array}$$

(12) $$\begin{array}{c} \text{Specificity}=\frac{\left|b\cap d\right|}{\left|b\right|}, \end{array}$$

(13) $$\begin{array}{c} \text{Dice}=\frac{\left|a\cap c\right|}{\left|\left.a\right|+\left|c\right|\right./2}. \end{array}$$

In the equations, *a*, *b*, *c*, and *d* represented the real ICH area (including the hematoma area), the ICH area (the hematoma area included) segmented by the intelligent algorithm, the real non-ICH area, and the non-ICH area segmented by the intelligent algorithm, respectively.

### 2.5. Observation Indexes and Grouping

The observation indexes included blood indexes and serological observation indexes of the patients in the two groups. Blood pressure indexes included diastolic blood pressure (DBP), systolic blood pressure (SBP), and mean arterial pressure (MAP). Serological observation indexes included low density lipoprotein (LDL), high density lipoprotein (HDL), total cholesterol (TC), triglyceride (TG), white blood cell count (WBC), hemoglobin concentration (HGB), red blood cell count (RBC), absolute neutrophil count (ANC), absolute lymphocyte count (ALC), and neutrophil-to-lymphocyte ratio (NLR).

### 2.6. Statistical Methods

Statistical software SPSS19.0 was used to process the experimental data. The measurement data were expressed as mean ± standard deviation ($\bar{x}\pm s$). The comparison in average values between groups was performed by *t* test. The enumeration data were expressed by percentage (%), and analyzed by *χ*^2^ test. *P* < 0.05 indicated that the difference was statistically significant.

## 3. Results

### 3.1. General Data and Results of the Two Groups of Patients

Figure 1 displays the comparison charts of the basic data of patients in the two groups. It was shown that there was no significant difference in the average age and gender ratio between the two groups (*P* > 0.05). The SBP, DBP, and MAP of patients in the observation group were significantly higher than those of the control group, showing the statistically significant differences (*P* < 0.05).

### 3.2. Cerebral CT Image Analysis of ICH Patients under Intelligent Segmentation Algorithm

The brain CT images before and after intelligent algorithm processing are presented in Figure 2 in the two groups of patients. It was observed that the CT images of the ICH patients processed by the intelligent segmentation algorithm were clearer, and the identification of the lesion edge was also easier.

### 3.3. CT Image Quality Evaluation under Intelligent Segmentation Algorithm

Figure 3 shows the comparisons of evaluation indexes of the image processing quality under the intelligent segmentation algorithm. The results suggested that the sensitivity, specificity, and accuracy (Dice) of CT images processed by the intelligent segmentation algorithm were 0.894, 0.898, and 0.930, respectively.

### 3.4. Comparison of CT Imaging Features between the Two Groups

The comparison of edema/hematoma volume in two CT images of patients between two groups is presented in Figure 4. The results suggested that the difference of the edema volume between the initial CT examination and follow-up CT examination of the patients with ICH was significantly greater in the observation group than that in the control group. Thus, the early edema enlargement degree in the observation group was significantly greater than that in the control group, with the statistically significant difference (*P* < 0.05). Similarly, the early hematoma enlargement in the observation group was also significantly greater than that in the control group, and the difference was statistically significant as well (*P* < 0.05).

Figure 5 shows the comparison of the relative edema volume of the CT images of two examinations between the two groups. As shown from the figure, the relative edema volumes of the observation group and the control group were 0.912 and 1.017, respectively, suggesting that the difference between the two groups of data was statistically significant (*P* < 0.05).

Figure 6 displays the comparison of various signs of CT images of patients in the two groups. Among the signs of CT images in ICH patients, the incidences of blend sign, low density sign, and island sign in the observation group were significantly higher than those in the control group, indicating that the differences were statistically significant (*P* < 0.05). There was no significant difference in the incidence of satellite sign between groups (*P* > 0.05).

### 3.5. Results of Serological Indexes of Patients in Two Groups

The comparison of the results of serological indexes of the patients in the two groups is displayed in Figure 7. According to the results, ALC, NLR, and HGB of the observation group were 6.23 × 109/L, 0.99 × 109/L, and 6.29 × 109/L, respectively. ALC, NLR, and HGB of the control group amounted to 6.08 × 109/L, 1.43 × 109/L, and 4.25 × 109/L, respectively. The differences in ALC, NLR, and HGB between the patients in the two groups were remarkable with statistical meaning (*P* < 0.05). In contrast, there were no significant differences in LDL, HDL, TC, TG, ANC, and RBC between the patients in the two groups (*P* > 0.05).

## 4. Discussion

In recent years, there are several reports that the amount and location of hematoma at the beginning of intracerebral hemorrhage were considered to be closely related to the prognosis of spontaneous intracerebral hemorrhage, which could be used as an effective predictive factor [20]. An intelligence segmentation algorithm was introduced to process cerebral CT images of patients with cerebral hemorrhage. After that, the application values of cerebral CT images in predicting early edema enlargement among patients with cerebral hemorrhage were assessed by measuring intracranial edema volume, hematoma volume, relative edema volume, and the frequency of the occurrence of various CT image signs. In addition, the reliability of serological indexes in the prediction of early edema enlargement was investigated. The research result revealed that the mean of sensitivity, specificity, and correctness rate of the used FCM intelligence segmentation algorithm in the segmentation of cerebral CT images of patients with cerebral hemorrhage reached 0.894, 0.898, and 0.930, respectively. CT images of patients with cerebral hemorrhage processed by intelligence segmentation algorithm became clearer with easier recognition of lesion edge. The results suggested that the segmentation of CT images processed by the intelligence segmentation algorithm was more precise compared with original CT images. In addition, the division of edema areas in CT images and the recognition of various signs of patients with cerebral hemorrhage became more simple and efficient.

What is more, hematoma was defined as the first increase of hematoma volume by 12.5 mL or over 33% during the subsequent CT scan for patients with intracranial hemorrhage in most studies. The factors causing hematoma enlargement among patients with cerebral hemorrhage included primary hypertension, cerebral amyloid angiopathy, diabetes, and abnormal coagulation [21]. Considerable studies proved that hematoma enlargement among patients with cerebral hemorrhage was remarkably correlated with neurological deterioration, poor prognosis, and death. If hematoma volume was enlarged by 10%, fatality would increase by 5%. No matter how hematoma enlargement was defined, there was a clear degree-response relationship between the enlarged volume as well as functional prognosis and fatality [22]. The comparison of hematoma between the patients in the two groups demonstrated that early edema enlargement and hematoma enlargement of patients in the observation group were more apparent than those in the control group, and the differences were remarkable with statistical meaning (*P* < 0.05). The relative edema volumes of the patients in the observation group and the control group were 0.912 and 1.017, respectively. The differences of the data between the two groups were significant with statistical meaning (*P* < 0.05).

The observation on the signs of CT images of patients with cerebral hemorrhage showed that the incidence of blend sign, low density sign, and stroke of the observation group was obviously higher than those of the control group with significant differences and statistical meaning (*P* < 0.05). It could be inferred that the blend sign, low density sign, and stroke of CT images of patients with cerebral hemorrhage could be used as the indicators of predicting early edema enlargement. The increase in water content in patient cerebral tissue and the enlarged cerebral volume resulted in increased intracranial pressure. Displacement of cerebral middle line and cerebral hernia caused the changes in the corresponding signs. The intracranial situation of patients after cerebral hemorrhage could be effectively detected by observing CT image characteristics to avoid further hematoma enlargement in time. Relevant studies suggested that patients with intracranial hemorrhage could be effectively intervened by analyzing the potential correlation between the specificity of hematoma among patients with spontaneous intracranial hemorrhage in CTA and CT and early hematoma enlargement during the clinical treatment of patients with cerebral hemorrhage to reduce fatality and improve prognosis [23].

The serological indexes of patients in the two groups showed that the ALC, NLR, and HGB of the observation group were 6.23 × 109/L, 0.99 × 109/L, and 6.29, respectively; those of the control group were 6.08 × 109/L, 1.43 × 109/L, and 4.25, respectively. The differences in ALC, NLR, and HGB between the two groups were significant (*P* < 0.05). No significant difference was found in LDL, HDL, TC, TG, ANC, and RBC between the two groups (*P* > 0.05). This showed that the serological indexes of ALC, NLR, and HGB in patients with ICH are significantly different between groups with or without hematoma enlargement. They could be taken as early predictors of hematoma enlargement after ICH, which was consistent with the findings of Cai et al. [24]. Both the researches confirmed the potential of the number of lymphocytes in the blood in the early prediction of hematoma enlargement after ICH. Some studies have suggested that the increase of WBC and ANC in ICH patients is one of the risk factors for island sign on CT images, while the increase of ALC is one of the protective factors of island sign. After the occurrence of ICH, the higher the WBC and ANC, the lower the ALC, the higher the NLR, and the higher the incidence of the island sign; the risk of early hematoma enlargement may also increase [25]. It has been reported that the relationship between the ANC and hematoma enlargement in patients with ICH may be caused by the destruction of peripheral blood vessels by neutrophils secreting metalloproteinases. Besides, the systemic inflammatory response after ICH may also lead to an increase in WBC and ANC as well as a decrease in ALC [26]. Another report indicates that upregulation of tissue factor expression in neutrophils can promote the formation of thrombin and affect the activity of the tissue factor inhibitory pathway [27]. In brief, most of the current studies have confirmed the application value of ANC and NLR in predicting hematoma enlargement after ICH.

## 5. Conclusion

Based on intelligence segmentation algorithm, cerebral CT images were processed to assess its application values in early edema enlargement among patients with cerebral hemorrhage. The results demonstrated that the cerebral CT images processed by intelligence segmentation algorithm showed high sensitivity, specificity, and correctness rate. Besides, ALC, NLR, and HGB of patients with cerebral hemorrhage also could predict hematoma enlargement after cerebral hemorrhage. Nevertheless, there were still some disadvantages in the research. For example, the included sample size was small. The predicative factors of hematoma enlargement among patients with cerebral hemorrhage with different stages and sites were discussed. In addition, the used algorithm had low noise resistance and the complexity of the algorithm affected image segmentation rate to some extent, which needed to be further optimized in future. To conclude, intelligence segmentation algorithm-based cerebral CT image and some serological indicators (ALC, NLR, and HGB) showed good clinical predictive values in hematoma enlargement after cerebral hemorrhage among patients, which provided certain reference values for the prediction of early hematoma enlargement among patients with cerebral hemorrhage.

## Figures and Tables

**Figure 1:** Comparison of the basic data of the two groups. (a–c) The comparisons of the average age, gender distribution, and blood pressure indexes of patients in the two groups, respectively. ^∗^Compared with control group, *P* < 0.05.

**Figure 2:** Comparison of cerebral CT images before and after being processed by intelligent algorithm. (a and c) The original cerebral CT images of patients in the observation group and the images processed by intelligence segmentation algorithm, respectively (the patient was a male aged 71). (b and d) The original cerebral CT images of patients in the control group and the images processed by intelligence segmentation algorithm (the patient was a female aged 74).

**Figure 3:** Comparison of evaluation indexes of image processing quality under intelligent segmentation algorithm. (a–c) The comparison charts of Dice value, sensitivity, and specificity, respectively. M1, M2, M3, M4, and M5 represented the 1^st^, 2^nd^, 3^rd^, 4^th^, and 5^th^ algorithm tests, respectively.

**Figure 4:** Comparison of edema/hematoma volume in CT images of patients between two groups. ^∗^Compared with control group, *P* < 0.05.

**Figure 5:** Comparison of relative edema volume in two CT examinations of two groups. ^∗^Compared with control group, *P* < 0.05.

**Figure 6:** Comparison of signs in two CT images of patients between two groups. ^∗^Compared with those of the control group, *P* < 0.05.

**Figure 7:** Comparison of serological indexes of patients between the two groups. (a) The comparison chart of ANC, ALC, and NLR. (b) The comparison chart of RBC and HGB, (c) The comparison of the cholesterol indexes of patients in the two groups. ^∗^Compared with the data of the control group, *P* < 0.05.

## Data Availability

The data used to support the findings of this study are available from the corresponding author upon request.
